This article has been retracted.

# Symptom Experienced Three Years after Liver Transplantation under Immunosuppression in Adults

**DOI:** 10.1371/journal.pone.0080584

**Published:** 2013-11-18

**Authors:** Chaoying Wang, Genshu Wang, Huimin Yi, Jianling Tan, Chi Xu, Xiaocui Fang, Yang Yang, Hua Li, Qier Chen, Guihua Chen

**Affiliations:** 1 Nursing School, the First Affiliated Hospital of Chongqing Medical University, Chongqing, China; 2 Department of Hepatic Surgery, The Third Affiliated Hospital of Sun Yat-Sen University, Guangzhou, China; 3 School of Nursing, Sun Yat-sen University, Guangzhou, China; UNIFESP Federal University of São Paulo, Brazil

## Abstract

**Background & Aims:**

Immunosuppression-related symptom experience has not been covered thoroughly in long-term liver transplant recipients. The aim of this study was to assess the symptom experience of immunosuppressive therapy three years after liver transplantation and to correlate it with adherence to medications and sociodemographic or disease-related characteristics.

**Methods:**

This study included 94 liver transplant recipients who had survived for more than 3 years after liver transplantation. Symptom experience was measured by the 59-Item Modified Transplant Symptom Occurrence and Symptom Distress Scale (MTSOSD-59R) at the outpatient visits. Adherence to immunosuppressive drugs was assessed using the Basel Assessment of Adherence with Immunosuppressive Medication Scale (BAASIS).

**Results:**

Itching, concentration or memory problems, and fatigue were the three most frequent or most distressing symptoms. Factors significantly associated with a higher level of symptom frequency and distress were 3- to 5-year time cohort (i.e., time post-transplantation), and younger age. At the item level, concentration or memory problems were the most frequent and distressing symptoms in the 3- to 5-year time cohort. Itching was the most frequent and distressing symptom in the 5- to 9-year time cohort. Finally, relationship was found between symptom experience and nonadherence to immunosuppressive drugs.

**Conclusions:**

Symptoms related to physical complaints or impairments were more often perceived and more distressing for liver transplant recipients 3 years after transplantation. Furthermore, the 3- to 5-year time cohort and younger age were associated with a higher degree of perceived symptom occurrence and symptom distress. Finally, recipients who perceived higher levels of symptom frequency and symptom distress reported higher levels of nonadherence.

## Introduction

The first liver transplantation (LT) in China was carried out in the 1970s. Thanks to better surgical techniques and care, survival outcomes after LT in adult recipients in China have gradually improved to a 3-year survival rate of 60.1% and 5-year survival rate of 55.6% [1]. As long-term survival for this particular operation has now improved, a simple focus on objectives clinical outcomes after LT cannot provide a sufficient evaluation of the results of medical treatment after LT any more. Therefore, attentions have been gradually moved to the patients’ subjective experiences [2-4].

Subjective outcomes are collectively referred to as ‘patient reported outcomes’ (PROs) [2]. PROs may help us evaluate the utility of transplantation and the effect of new drugs or devices employed after transplantation [2,3,5,6]. Symptom experience and medication adherence are two major aspects of PROs to LT recipients.

LT recipients require lifelong treatment with immunosuppressive medications, such as tacrolimus , sirolimus , mycophenolate mofetil and cyclosporine, which are associated with a broad range of immunosuppression-related side effects [7-9]. Side effects based on biochemical model, such as hypertension, diabetes, and renal dysfunction, have concerned physicians. Nevertheless, some other side effects that are subjective experienced by LT recipients, including itching, fatigue, lack of energy, and trembling hands, may be very disturbing and have not been given sufficient attention. These symptoms can influence LT recipients’ medication adherence and quality of life [10-14]. Therefore, careful assessment and management of recipients’ perceived symptom experience associated with immunosuppressant-related side effects is crucial to formulating symptom management strategies that may help to reduce the symptom-related burden, promote medication adherence, and provide long-term recipients with a better quality of life after transplantation. 

Symptom experience refers to the recipients’ subjective experience of immunosuppressant-related adverse effects. It involves two parallel but interrelated concepts: symptom occurrence and symptom distress [15]. Symptom occurrence (cognitive pathway of symptom experience) is described as the frequency, severity, and duration of a given symptom perceived by an individual [15]. Symptom distress (emotional pathway of symptom experience) demonstrates how recipients are influenced daily by these symptoms [15]. Many of the most frequent symptoms may not be perceived as the most distressing symptoms, and vice versa; therefore, the distinction between these two concepts is of prime importance. 

The period of time after transplantation is one determinant of the perception of symptom experience [13,16-19]. However, few studies have evaluated the symptom experience after LT, especially in recipients who have survived 3 years or more after LT. The immunosuppressant protocol of these recipients are substantially different from recipients who survived a shorter period. Some other determinants of symptom experience among patients who have undergone other organ transplantations are gender [10,13,18,20,21], age [13,19], pre-transplant diagnosis [22], and immunosuppressant protocol [23]. A link between symptom experience and nonadherence has been found in patients who have undergone other types of organ transplantations, such as heart, renal, and lung transplantations [13,17,24-26]. However, scarce data currently exists on the relationship between symptom experience and adherence to immunosuppressive drugs in LT recipients, especially those who have survived for 3 years or more after LT.

Thus, the aims of this study were to (1) evaluate the symptom experience associated with immunosuppressive drugs in adult LT recipients surviving for more than 3 years after LT, (2) examine the influence of gender, age, time after LT, employment status, marital status, pretransplant diagnosis, and immunosuppressant protocol on symptom experience, and (3) explore the possible relationship between symptom experience and adherence to immunosuppressive medications.

## Materials and Methods

### Design and sample

A cross-sectional study was adopted. During the course of 3 months, adult recipients of the Third Affiliated Hospital of Sun Yat-sen University in Guangzhou, China were recruited to this study during their protocol post-LT outpatient visits. Inclusion criteria for the study were: (1) 18 years or older at the time of LT, (2) underwent LT at least 3 years prior to study inclusion, (3) able to understand and communicate in Chinese, and (4) provided written informed consent. Recipients were excluded if they (1) had undergone retransplantation or were on the waiting list for a retransplantation, (2) had psychiatric or brain disease, or (3) could not be assessed because of illness such as a terminal illness or hospitalization for a serious condition. A total of 98 LT recipients were asked to enroll in the study. Two recipients refused and two recipients did not complete the questionnaire, yielding a convenience sample of 94 subjects. Comparison of their characteristics (gender, *P* = 0.93; age, *P* = 0.79; time post-transplantation, *P* = 0.06; and immunosuppressant protocol, *P* = 0.13) with those of 238 eligible recipients in the hospital showed no statistically significant differences. 

### Measurements

#### Symptom experience

Symptom experience associated with the immunosuppressive regimen was measured by the 59-Item Modified Transplant Symptom Occurrence and Symptom Distress Scale (MTSOSD-59R), which is exclusively used to assess the patient’s appraisal of symptoms associated with side effects of immunosuppressive therapy [3,28]. This instrument is the latest updated version at the time of the present study and based on the 29- and 45-item versions by Moons et al [10,27], and had been translated into 11 different languages as a useful instrument. Further, MTSOSD-59R focus narrowly on the adverse effects of immunosuppressive medication in all types of transplantation with an assessment of psychometric properties and can effectively capture many subjective symptoms related to immunosuppressive drugs that may be experienced by organ transplant recipients instead of those that can only be distinguished by objective tests [28]. Lastly, the ability of the MTSOSD-59R to distinguish between symptom experience of recipients on immunosuppressive regimens and that of patients not receiving immunosuppressive drugs demonstrates the discriminant validity [28]. The above points accordingly illustrate that the data, namely the studied symptoms collected by MTSOSD-59R is closely related to the use of immunosuppressive drugs.

Each item represented a symptom that was scored in terms of both symptom occurrence and symptom distress. The instrument differed in gender for one item: impotence for men and menstrual problems for women [28]. The items were assessed on a 5-Likert scale, ranging from 0 (never occurring) to 4 (always occurring) for symptom occurrence and from 0 (not at all distressing) to 4 (extremely distressing) for symptom distress [28]. To prevent inclusion of anticipatory distress, the response on that item of the symptoms was converted to missing value when the symptoms reported by the patient as never occurring on the symptom occurrence scale (score=0) but as distressing on the symptom distress scale. For this Chinese population, the instrument was translated into Chinese and back into English following a standard translation protocol [29]. Content validity was determined by two eminent surgeons who worked with LT recipients and three nursing specialists who worked in the School of Nursing of Sun Yat-sen University. Cronbach’s alpha for symptom occurrence and symptom distress were 0.92 and 0.94, respectively. The test-retest reliability for each was both 0.96.

#### Adherence to immunosuppressive drugs

Self-reported adherence to immunosuppressive regimens was detected using the Basel Assessment of Adherence with Immunosuppressive Medication Scale (BAASIS), developed by The Leuven Basel Adherence Research Group [30]. This instrument comprised a four-item validate questionnaire to assess medication adherence (dose-taking, drug holidays, timing deviation of >2 h, and dose reduction). One item evaluated the persistence of immunosuppressive drug-taking, and a 10-cm visual analog scale (VAS) was used to assess overall medication adherence [30]. All items that evaluated adherence started with a YES/NO question. Any self-reported “YES” (nonadherence) on any of the items was considered as nonadherence. Alternatively, answering “NO” on all of the items was considered as adherence. On the persistence item, LT recipients who answered “YES” were considered to be non-persistent. The VAS score was expressed as a percentage with no defined cut-off for nonadherence [30]. The instrument was translated into Chinese and back into English following a standard translation protocol [29]. Content validity was determined by five specialists. Cronbach’s alpha for all items was 0.71, and the test-retest reliability was 0.95.

#### Demographic and clinical variables

Demographic characteristics included age, gender, marital status, education level, employment status, time since LT, and immunosuppressive drug protocol. The time after LT was arbitrarily divided into a 3- to 5-year time cohort and a 5- to 9-year time cohort according to the survival classification method.

### Ethics statement

This study was approved by the ethics committee of the Third Affiliated Hospital of Sun Yat-sen University in Guangzhou, China. Written informed consent was obtained prior to data collection.

### Procedures

A pilot test involving 15 LT recipients in the outpatient LT department was carried out, and the test-retest reliability was measured at 4-week intervals before the formal investigation. Eligible recipients were asked to participate in this study during their regular outpatient clinical visits after LT. The investigator instructed them how to fill out the MTSOSD-59R and BAASIS, especially emphasizing the necessity and significance of bearing it in mind that only the symptoms associated with immunosuppressive therapy are supposed to be included when fill out the MTSOSD-59R. The recipients were asked to complete the questionnaires on the spot. Completeness was checked, and the recipients were asked to complete missing data if necessary. Clinical data were collected from the medical files.

### Statistical analysis

Data were analyzed using the statistical software SPSS, version 16.0. Frequency, mean, standard deviation, median, and interquartile range (P25; *P*75) were used for statistical descriptions depending on the distribution. For two-group comparisons, the *t*-test, Mann-Whitney *U*-test, chi-squared or correction for continuity, and Fisher’s exact probability tests were used. Correlations between symptom experience and medication adherence were tested by Spearman’s correlation.

Ridit analysis, a sensitive method for ordinal data, was used to analyze symptom experience. A ridit refers to a probability measure of an identified distribution. The ridit of a (sub)sample will always be compared with the ridit of the chosen reference group. According to the instructions by Moons [26], the reference group for comparison among symptoms in this study was determined using the occurrence distribution of the whole sample over all items and over the respective symptoms for comparison between the 3- to 5-year time cohort and the 5- to 9-year time cohort at the item level. The level of significance was set at *P* < 0.05.

## Results

### Patient group

The demographic and clinical characteristics of the recipients are listed in Table 1. A total of 94 eligible recipients with a mean age of 51.4 years (SD, 11.0; range, 28–74) were included in the study. The median time post-LT was 5.1 years (interquartile range, 2.77; range, 3–9). Most of the subjects were men (90.4%) and were married (95.7%), and 56 (59.6%) had attained a high school or higher education. The percentage of employed subjects (56.4%) was higher than that of unemployed subjects (40.4%). The primary liver disease was hepatocellular carcinoma (36.2%). Most of the recipients were undergoing treatment with a tacrolimus-based immunosuppressive regimen (88.3%).

**Table 1:** Comparison of demographic and clinical characteristics between the different time cohorts.

**Variable**	**Total sample (n=94)**	**3- to 5-year time cohort (n=46**)	**5- to 9-year time cohort (n=48**)	***P* Value**
Age (yr, M±SD)	51.4±11.0	50.5±10.3	52.3±11.8	NS
Time after transplantation (yr, M±SD)	4.6±1.5			
Gender				NS
Male	85 (90.4)	41 (89.1)	44 (91.7)	
Female	9 (9.6)	5 (10.9)	4 (8.3)	
Employment status (n/%)				NS
Unemployed	41 (43.6)	21 (45.7)	20 (41.7)	
Employed	53 (56.4)	25 (54.3)	28 (58.3)	
Marital status (n/%)				NS
Married	90 (95.7)	43 (93.5)	47 (97.9)	
Never married/Divorced	4 (4.3)	3 (6.5)	1(2.1)	
Education level (n/%)				NS^a^
≤Junior high school	38 (40.4)	19 (41.3)	19 (39.6)	
≥Senior high school	56 (59.6)	27 (58.7)	29 (60.4)	
Primary liver disease (n/%)				NS^b^
Hepatocellular carcinoma	34 (36.2)	20 (43.5)	14 (29.2)	
Cirrhosis	33 (35.1)	13 (28.3)	20 (41.7)	
Hepatitis B	25 (6.4)	12 (26.1)	13 (27.1)	
others	2 (2.2)	1 (2.2)	1 (2.0)	
Immunosuppressive drugs (n/%)				0.03
Tac-based regimens	83 (88.3)	44 (95.7)	39 (81.3)	
Tac monotherapy	58 (61.7)	29 (63.0)	29 (60.4)	
Tac+SRL	6 (6.4)	4 (8.7)	2 (4.2)	
Tac+MMF	19 (20.2)	11 (23.9)	8 (16.7)	
Others	11 (11.7)	2 (4.3)	9 (18.8)	
CsA monotherap	2 (2.1)	0	2 (4.2)	
MMF monotherapy	4 (4.3)	0	4 (8.3)	
SRL monotherapy	2 (2.1)	2 (4.3)	0	
CsA+MMF	3 (3.2)	0	3 (6.3)	

Tac, tacrolimus; SRL, sirolimus; MMF, mycophenolate mofetil; CsA, cyclosporine

a Others were deleted

b Tac-based regimens vs. others

A comparison of the demographic and clinical characteristics between the different time cohorts post-LT is illustrated in Table 1. This table shows that different time cohort subjects shared the majority of the characteristics, although the ratio of tacrolimus-based immunosuppressive regimen utilization was higher in the 3- to 5-year time cohort than in the 5- to 9-year time cohort.

### Symptom experience

#### Overall ridit

Measured by MTSOSD-59R, all subjects demonstrated perceived immunosuppression-related symptoms with a median of 7 out of 59 (range, 2–43) and distress with a median of 4 out of 59 (range, 1–43). Comparison of the occurrence (*P* = 0.005) and distress of symptoms (*P* = 0.001) between genders revealed significant differences. These differences were also reported between the two time cohorts (*P* = 0.004 and *P* = 0.005). Specially, female gender and the 3- to 5-year time cohort reported higher levels of symptom frequency and distress. Symptom occurrence (*P* < 0.001) and symptom distress (*P* < 0.001) were significantly higher in younger than older subjects. Differences among marital status and primary liver diseases showed no statistical significance. Recipients who were employed reported a higher level of symptom occurrence (*P*<0.001), and this discrepancy was shared by recipients on the tacrolimus-based regimens (*P* = 0.02) (Table 2).

**Table 2:** Comparison of symptom occurrence and symptom distress based on recipient characteristics.

**Variable**	**SO ridit**	***t/χ2***	***P* Value**	**SD ridit**	***t/χ2***	***P* Value**
Gender		-2.783	0.005		-3.378	0.001
Male	0.495			0.471		
Female	0.511			0.500		
Time after transplantation (yr)		2.846	0.004		2.849	0.005
3-	0.507			0.480		
5-9	0.493			0.468		
Age (yr)		28.470	<0.001		19.301	<0.001
28-	0.555			0.512		
40-	0.490			0.468		
50-	0.496			0.469		
60-	0.485			0.464		
70-74	0.463			0.444		
Primary liver disease (n/%)		1.613	NS		1.876	NS
Hepatocellular carcinoma	0.494			0.467		
Cirrhosis	0.501			0.478		
Hepatitis B	0.507			0.477		
others	0.490			0.468		
Employment status (n/%)		4.210	<0.001		1.194	NS
Unemployed	0.488			0.477		
Employed	0.509			0.484		
Marital status (n/%)		-1.761	NS		0.892	NS
Married	0.500			0.474		
Never married/Divorced	0.525			0.484		
Immunosuppressive drugs		2.301	0.020		0.459	NS
Tac-based regimens	0.502			0.475		
Others	0.498			0.471		

SO, symptom occurrence; SD, symptom distress

#### Item scores

In terms of analysis on the item level of all subjects’ scores, the ten most frequent or distressing symptoms among all LT recipients who had survived for more than 3 years are illustrated in Table 3. The symptom occurrence and symptom distress distributions of all items are shown in Figures 1 and 2, respectively. Itching, concentration or memory problems, and fatigue were the three most frequent and distressing symptoms. Nine symptoms were both the most frequent and distressing, although their rank orders were not identical.

**Table 3:** Ten most frequent or distressing symptoms in all subjects.

**Rank order**	**Symptom occurrence**	**Ridit**	**Symptom distress**	**Ridit**
1	Itching	0.650	Itching	0.587
2	Concentration or memory problems	0.642	Concentration or memory problems	0.584
3	Fatigue	0.614	Fatigue	0.575
4	Sores on lips or in mouth	0.603	Diarrhea	0.571
5	Dizziness	0.599	Sleep difficulties	0.556
6	Sleep difficulties	0.587	Joint pain	0.551
7	Diarrhea	0.587	Sores on lips or in mouth	0.541
8	Lack of energy	0.559	Dizziness	0.540
9	Joint pain	0.552	Headache	0.531
10	Nightmares	0.547	Lack of energy	0.526

**Figure 1:** Distribution of symptom occurrence among all items.

**Figure 2:** Distribution of symptom distress among all items.

The rank order of the 10 most frequent symptoms reported by the 3- to 5-year time cohort and 5- to 9-year time cohort revealed that these two time cohorts shared 7 of the 10 most frequent symptoms, namely concentration or memory problems, itching, dizziness, sleep difficulties, fatigue, sores on the lips or in the mouth, and diarrhea (Table 4, Table 5). Concentration or memory problems (0.65) were the most frequently perceived symptoms in the 3- to 5-year time cohort, while itching (0.66) was the most frequently perceived symptom in the 5- to 9-year time cohort. Comparison on the item level demonstrated higher ridit for redness of the face or neck (*P* = 0.02) and muscle cramping (*P* = 0.04) in the 3- to 5-year cohort than in the 5- to 9-year cohort. 

**Table 4:** Rank order of the 10 most frequent symptoms perceived by the two time cohorts.

**Rank order**	**3- to 5-year time cohort symptom**	**Ridit**	**5- to 9-year time cohort symptom**	**Ridit**
1	Concentration or memory problems	0.652	Itching	0.659
2	Itching	0.641	Fatigue	0.654
3	Dizziness	0.629	Concentration or memory problems	0.632
4	Sleep difficulties	0.626	Diarrhea	0.595
5	Fatigue	0.623	Sores on lips or in mouth	0.577
6	Sores on lips or in mouth	0.621	Headache	0.575
7	Joint pain	0.602	Dizziness	0.569
8	Diarrhea	0.579	Back pain	0.558
9	Restlessness/nervousness	0.571	Trembling hands	0.553
10	Increased thirst	0.571	Sleep difficulties	0.551

**Table 5:** Rank order of the 10 most distressing symptoms perceived by the two time cohorts.

**Rank order**	**3- to 5-year time cohort symptom**	**Ridit**	**5- to 9-year time cohort symptom**	**Ridit**
1	Concentration or memory problems	0.588	Itching	0.600
2	Itching	0.573	Concentration or memory problems	0.588
3	Sores on lips or in mouth	0.571	Sleep difficulties	0.542
4	Sleep difficulties	0.569	Lack of energy	0.540
5	Joint pain	0.566	Joint pain	0.536
6	Dizziness	0.543	Dizziness	0.535
7	Headache	0.534	Fatigue	0.534
8	Increase sweating	0.525	Back pain	0.531
9	Lack of energy	0.518	Sores on lips or in mouth	0.527
10	Anxiety	0.513	Restless/nervousness	0.505

The rank order of the 10 most distressing symptoms reported by the two time cohorts after LT is shown in Table 4. Seven symptoms were among the 10 most distressing symptoms in both time cohorts: concentration or memory problems, itching, sores on the lips or in the mouth, sleep difficulties, joint pain, dizziness, and lack of energy. Concentration or memory problems (0.59) were the most distressing symptoms in the 3- to 5-year cohort, and itching (0.60) was the most distressing symptom in the 5- to 9-year cohort. Comparison of the two time cohorts at the item level revealed that increased sweating (*P* = 0.03), redness of the face or neck (*P* = 0.007), and sensitivity to light (*P* = 0.02) were significantly more distressing in the 3- to 5-year time cohort. Only hearing loss (*P* = 0.02) was significantly more distressing in the 5- to 9-year time cohort. 

### Adherence to immunosuppressive drugs

The prevalence of adherence to immunosuppressive drugs as assessed by the BAASIS revealed that 39.4% of LT recipients who had survived for more than 3 years were nonadherent. Nonadherence to timing of medication was found in 33.0% of recipients, which was the worst domain of medication adherence. Approximately 16.0% of recipients reported that they missed at least one dose, but only 1.1% of recipients changed doses without the doctor’s permission. No recipients stopped taking their medications completely within the last year.

### Correlation between symptom experience and adherence to immunosuppressive drugs

A positive correlation was found between symptom occurrence and nonadherence to immunosuppressive medications (*r* = 0.282, *P* = 0.006). The same correlation was found for symptom distress (*r* = 0.284, *P* = 0.006). Recipients who perceived a higher level of symptom frequency and symptom distress reported a higher level of nonadherence.

## Discussion

To date, this is the first study to assess symptom experience and its correlation with adherence to immunosuppressive medications in LT recipients who have survived for 3 years or more. Because immunosuppressive doses have decreased and immunosuppressive protocols have changed over time, the post-LT time may affect symptom occurrence. Long-term (≥-year) post-LT symptom experience may therefore differ from that among short-term recipients. 

In terms of quality of life, adherence to immunosuppressive mediations, and evaluation of medical care, an understanding of patients’ assessment of immunosuppressant-related adverse effects is of utmost importance. Because patients’ perceptions of symptom experience after LT differ from those of health care specialists, an understanding of patients’ perceptions may help to improve clinical outcomes of conditions such as hypertension, diabetes mellitus, and renal damage.

The present study demonstrated that itching, concentration or memory problems, and fatigue were the three most frequent and distressing symptoms. The majority of the 10 most frequent or distressing symptoms among all subjects were physical symptoms or impairments [13], such as fatigue, lack of energy, or joint pain. This finding is not consistent with the findings of previous studies showing that symptoms related to body image changes (e.g., moon face [13,27,31], increased hair growth [26,27,31,32], bruises [16,27] and changed facial features [16,19]) and symptoms related to psychological distress (e.g., mood swings [10,32] and anxiety [19]) were the 10 most frequent or distressing symptoms. In contrast, the 10 most frequent or distressing symptoms in these previous studies were the least frequent or distressing symptoms in the present study. The present results may be related to the immunosuppressive protocol. For example, symptoms such as moon face, a changed facial appearance, and bruises were the most frequently occurring or distressing symptoms perceived by recipients taking cyclosporine-based regimens [33] or corticosteroids [23]. However, in this study, 88.3% of recipients were on a tacrolimus-based regimen, consistent with the findings of Moons et al [10]. Another reason for these findings may be related to cultural differences; Chinese people are more likely to express physical rather than emotional discomfort [34]. A final reason for these findings may be that all subjects in the present study were LT recipients who had survived for 3 years or more. Previous studies found that symptoms such as joint pain, back pain, etc. became more frequent over time, while symptoms such as swollen gums and increased hair growth were less frequent 3 years after LT [17].

The results of this study also lend empirical support to a previous study by van Ginneken et al [35], who reported that fatigue, sleep difficulties, and lack of energy were interrelated. All 3 of these symptoms were among the 10 most frequent and distressing symptoms. Recipients with a feeling of daytime fatigue were more likely to increase their temporary inactivity or rest periods, which would affect their nighttime sleep quality and thus cause increased tiredness. In addition, recipients who felt daytime fatigue might be more likely to lack energy to return to work, possibly leading to isolation from society and increased sensitivity to physical discomfort. Symptom may occur in clusters [36]; therefore, health care specialists must view symptoms as influencing and being influenced by other symptoms when measuring symptom experience.

In the study, the most frequent symptoms were not necessarily the most distressing symptoms, as shown in previous studies [21,32]. This finding reveals the importance of separation of the concepts of occurrence and distress in relation to each item when assessing symptom experience.

Notably, the 3- to 5-year time cohort reported higher overall levels of symptom occurrence and symptom distress after LT compared with the 5- to 9-year time cohort. Because some side effects are dose-related, the immunosuppressive doses decreased over time, as did the gastrointestinal complaints [37], emotional burdens [18], and post-transplant diabetes-related symptoms [38]. Therefore, symptom occurrence and symptom distress were higher in the 3- to 5-year time cohort than in the 5- to 9-year time cohort.

As shown in previous studies, the present study revealed that symptom experience was influenced by age. Younger recipients had a higher level of symptom occurrence and distress compared with older recipients [10,13,19]. Younger recipients were often more active and experienced pressure from family and work, which may have affected their sensitivity to side effects. Furthermore, because of the relatively low basal metabolism rate (BMR) in older recipients, their immunosuppressive doses were lower than those of younger recipients, which may have impacted their symptom experience. These findings are consistent with those of Winsett et al [18].

The results of the comparison of symptom experience between genders were consistent with those of other related studies [10,13,19,27]. Women reported higher overall levels of both symptom occurrence and symptom distress. Psychosocial factors may result in a higher sensitivity to physical complaints in females [31]. In addition, females are more sensitive to the side effects of medications [39], which in turn might cause a higher level of symptom occurrence. However, given the limited data presented (only 9 females), more studies about gender differences would in need.

In a previous study, the relationship between the employment status and symptom experience was not found in renal transplant recipients [40], while this study showed that recipients who were employed might experienced a higher level of symptom occurrence. Those who did work may be charged with more social responsibility, and have higher level of stress. Further, recipients who were employed were more weak in terms of psychosocial adjustment [41]. The above points might illustrate the outcome.

A life-long successful immunosuppressive regimens is important in organ transplantation and depends on various factors such as adherence to immunosuppressive medications and quality of life [13,23]. Symptom experience can predispose recipients to nonadherence. As shown in a previous study by de Barros et al., who assessed medication nonadherence by interviewing renal transplant recipients [31], the present study revealed that recipients who reported higher levels of symptom occurrence and symptom distress were more likely to be nonadherent.

This study extends the findings of previous studies on the symptom experience of transplant recipients [10,21,26,27,31]. First, most previous studies used the 29- or 45-item MTSOSD scale, neither of which includes symptoms related to the newest immunosuppressants. Second, the subjects of this study were all recipients who had survived for 3 years or more. Third, ridit analysis was employed in the study. However, one must keep in mind that symptoms experienced by recipients may not be caused by immunosuppressive drugs directly. While the instrument is an internationally accepted standardized measure which intend to assess symptoms associated with the side-effects of the immunosuppressive regimens, some items may refer to symptoms of the underlying disease or other worsening conditions. Therefore, it should be checked further in future studies. In addition, the findings of this study are limited by the selection of one hospital sample in mainland China, which restricts its generalizability. Lastly, taking palliative medication may affect any correlation with immunosuppressive adherence, for it may relieve side effects of immunosuppressive drugs, and further research is needed to investigate the influence of palliative medication.

In conclusion, this study found that symptoms related to physical complaints or impairments were more often perceived and more distressing to LT recipients who had survived for 3 years or more. Furthermore, younger age and the 3- to 5-year time cohort were associated with a higher degree of perceived symptom occurrence and symptom distress. Finally, recipients who perceived a higher level of symptom frequency and symptom distress reported a higher level of nonadherence. The results of this study could be used to prepare the recipients for these symptoms so that they would consider them as ‘normal’ for this therapeutic intervention. In addition, identifying the factors which might be affected the symptom experience is important for offering them education and advice about the adverse effects caused by immunosuppressive therapy.
